The article "Application Research for Fusion Model of Pseudolabel and Cross Network" was published in 2022. Journal: Comput Intell Neurosci.

# Application Research for Fusion Model of Pseudolabel and Cross Network

**DOI:** 10.1155/2022/9986611

**Published:** 2022-05-19

**Authors:** Junying Gan, Bicheng Wu, Qi Zou, Zexin Zheng, Chaoyun Mai, Yikui Zhai, Guohui He, Zhenfeng Bai

**Affiliations:** Department of Intelligent Manufacturing, Wuyi University, Jiangmen, Guangdong 529020, China

## Abstract

Datasets usually suffer from supervised information missing and weak generalization ability in deep convolution neural network. In this paper, pseudolabel (PL) of Weakly Supervised Learning (WSL) was used to address the problem of supervised information missing, while Cross Network (CN) of Multitask Learning (MTL) was used to solve the problem of weak generalization ability in deep convolution neural network. In PL, the data of supervised information missing was predicted; thus, PL of the corresponding data was generated. In CN, PL data and labeled data were taken as two tasks to train together. Firstly, the labeled data was divided into training dataset and testing dataset, respectively, and image preprocessing was carried out. Secondly, the network was initialized and trained, and the model with high accuracy and good generalization was selected as the optimal model. Then, the optimal model was used to predict the unlabeled data and generate PL. Finally, the steps above were repeated several times to find a better optimal model. In the experiments of the fusion model of PL and CN, Facial Beauty Prediction was regarded as main task and the others as auxiliary tasks. Experimental results show that the model was suitable for multitask training of different tasks in different or similar datasets, and the accuracy of the main task of Facial Beauty Prediction reaches 64.76%, higher than the highest accuracy by conventional methods.

## 1. Introduction

In practical applications, datasets often suffer from incompletely or unclearly supervised information. However, deep learning models are still expected to obtain better results in the case of some tasks where sufficient and high-quality real labels are difficult to obtain. Thus, Weakly Supervised Learning (WSL) was proposed. It can train a deep learning model with strong generalization ability even if the data labels are not all true, which reduces the cost of data labeled annotation in Supervised Learning (SL) and saves manpower and resources. For this reason, WSL was applied in this paper to train the data. Reference [1] proposed pseudolabel (PL), which trained both labeled data and unlabeled data in a supervised way, and predicted unlabeled data to generate PL. Experimental results based on MNIST dataset were better than that by the other methods. Reference [2] replaced simple noise operation by innovative data augmentation methods, such as RandAugment and Back-Translation. Under the same training framework, experiments based on six languages and three visual tasks achieved good results. On IMDB Text Classification Dataset, only 20 labeled samples were used, and the accuracy was 95.8%, higher than that of the model trained on 25,000 labeled samples. Only 250 labeled samples were used in CIFAR-10 Dataset, and the accuracy was 94.57%. Reference [3] proposed MixMatch algorithm, by way of MixUp to estimate the low entropy label in data. The data included the unlabeled samples and mixed samples after data augmentation. The mixed samples included unlabeled data and labeled data. Through 250 labeled samples in CIFAR-10 dataset, the error rate was reduced four times from 38% to 11%. Reference [4] improved MixMatch algorithm by introducing distributed alignment and enhanced anchoring method. Only 250 labeled samples were used in CIFAR-10 dataset, and the accuracy was up to 93.73%. Among them, MixMatch used 4000 labeled samples to achieve the accuracy of 93.58%. Reference [5] used consistent regularization and PL to improve the performance of the model. Firstly, the model was used to generate PL for weak augmentation of unlabeled sample. Then, the strong augmentation of the same sample was input to train the model and predict PL. Only 250 labeled samples were used in CIFAR-10 dataset, and the accuracy was as high as 94.93%. On the 40 labeled samples, the accuracy was as high as 88.61%. Reference [6] proposed to explicitly estimate the prediction uncertainty during training to rectify the pseudolabel learning for unsupervised semantic segmentation adaptation. The uncertainty was involved into the optimization objective as the variance regularization to rectify the training. The regularization helped the model learn from the noisy label without introducing extra parameters or modules. Experimental results demonstrated that the competitive performance was achieved. Reference [7] proposed an uncertainty-guided noise resilience network, in which the confidence of the target domain samples to predict pseudolabels was explored.

The article "Application Research for Fusion Model of Pseudolabel and Cross Network" was published in 2022. Journal: Comput Intell Neurosci.

WSL can solve the problem of unlabeled data, but the effect by only using WSL was not ideal. Therefore, a learning paradigm combining WSL with Multitask Learning (MTL) was presented in this paper. MTL has been proved to be effective in solving computer vision problems [8]. For different tasks, the best sharing layer was often different, and there was no unified standard. An unsupervised scene adaptation method of learning from both labeled source data and unlabeled target data was proposed, in which memory regularization in vivo was presented to exploit the intradomain knowledge and regularize the model training, and the primary classifier and the auxiliary classifier were applied to reduce the prediction inconsistency without any extra parameters or external modules [9]. Reference [10] proposed a novel unsupervised domain adaptation framework based on an iterative self-training procedure, which could alternately generate pseudolabels on the target data and retrain the model with these labels. Reference [11] proposed Cross-Stitch Networks by activating the network for End-to-End Learning and then automatically deciding the shared layer, in which network with Cross Unit could learn the best combination of shared feature and independent feature representation, effectively solving the problem of not being able to make full use of relevant task information. Reference [12] proposed a new end-to-end Coattentive Multitask Convolutional Neural Network (CMCNN), which was composed of the Channel Coattention Module (CCAM) and the Spatial Coattention Module (SCAM). Functionally, the CCAM generated the channel coattention scores by capturing the interdependencies of different channels between FER and FLD tasks. The SCAM combined the max-pooling and average-pooling operations to formulate the spatial coattention scores.

The fusion model of WSL and MTL can solve the problem of supervised information missing of data labels and make use of relevant task information to improve the generalization ability of the model. Reference [13] proposed WILDCAT (Weakly Supervised Learning of Deep Convolutional Neural Networks), which aligned image regions to obtain spatial invariance and learn obvious local features by only using global image labels for training. This method focused on three main visual recognition tasks, including Image Classification, Weakly Supervised Object Localization, and Semantic Segmentation. In this paper, full convolution network to maintain spatial resolution, and Weakly Supervised Localization of different salient local features of the object were used. The network could recognize multiple local regions. Reference [14] aimed at the difficulty of collecting a large number of training datasets by manually marked labels and proposed to divide these weakly supervised source domain labels into several different but related subtask model, respectively. Reference [15] proposed to leverage these datasets using weakly supervised multitask learning to improve the generalization performance on each of them. Specifically, three multimodal affect recognition tasks were explored, including emotion recognition, sentiment analysis, and sarcasm recognition.

The article "Application Research for Fusion Model of Pseudolabel and Cross Network" was published in 2022. Journal: Comput Intell Neurosci.

In this paper, the fusion model of PL and Cross Network (CN) was presented. Facial Beauty Prediction was regarded as main task and the others as auxiliary tasks. WSL was used for supervised information missing. In deep convolution neural network, MTL was used for the weak generalization. PL can utilize the data without real label for network training, saving a lot of time and economic cost. In CN, the network with Cross Unit can learn the best combination of shared features and independent features. The fusion model of PL and CN can solve the problems of weak generalization ability and supervised information missing.

## 2. Design and Implementation of Fusion Model of PL and CN

The fusion model of PL and CN was shown in Figure 1. Firstly, the labeled dataset was divided into testing dataset and training dataset, in which training dataset was used for model parameter training, and the model with high accuracy and good stability was selected as the optimal model. Secondly, the unlabeled dataset was fed into the optimal model for PL prediction. So, the predictive model generated PL corresponding to the data. Thirdly, training dataset and PL dataset were fused, preprocessed and fed to single-task/multitask model to predict. Finally, testing dataset was used to test the accuracy of single-task/multitask model to find a better model with higher accuracy and better stability, which could be used as the next prediction model for the unlabeled dataset.

The classification network of fusion model of PL and CN mainly included two parts: PL data generation part and data cotraining part. In the PL data generation part, each network model was trained through the training dataset, and the optimal model with high accuracy and good stability was selected as PL generation model. The unlabeled data was input into the optimal model and the predictive value was output. Thus, the predictive value was PL of the corresponding data, and the unlabeled dataset was transformed into PL dataset. In the data cotraining part, PL data and training dataset were used to train each network model. Therefore, better comprehensive model was selected and used as the model to generate PL. The unlabeled data was input into the optimal model again to output the prediction, and the output value was PL of the corresponding data. The steps above were repeated several times until the end condition that the accuracy could not be improved was met. Each part of the model was discussed below.

### 2.1. Data Preprocessing

Figure 2 was the data preprocessing part, whose main task was to perform relevant processing on the samples, including data augmentation, rotation, and cropping operations. This operation facilitated the input and feature learning of the subsequent network. To solve the problem of few training samples, different data augmentation methods were applied to expand the sample number of training dataset, which was random clipping, random image flipping from left to right, and random image rotation. For normal multitask training process, samples with the same order of magnitude were used to train model and test model in each task. At the same time, the key work was deduplication, normalization, clipping, and rotation. Through the similar comparison algorithm, some images with high repeatability or low resolution were removed. At the same time, the images were cut to a uniform image resolution and normalized.

The article "Application Research for Fusion Model of Pseudolabel and Cross Network" was published in 2022. Journal: Comput Intell Neurosci.

### 2.2. PL Data Generation

Figure 3 was the specific process of PL data generation. The labeled dataset was divided into training dataset and testing dataset. Then, the training dataset was input into various models after data preprocessing, including VGG16 [15] and ResNet50 [16], Transfer Network based on VGG16, and ResNet50 with pretrained parameters. In the meantime, the model and hyperparameters were adjusted continuously to obtain a better model. According to the criterion of high accuracy and good stability on testing dataset, the optimal model was selected as the model of PL prediction. After data preprocessing, the unlabeled data was input into the optimal model and then predicted to generate PL. As a result, pseudolabeled dataset was generated.

### 2.3. Data Cotraining

Figure 4 was the specific process of data cotraining part, in which the labeled dataset and PL dataset were fused. After data preprocessing, they were input into various models, including VGG16 and ResNet50, Transfer Network based on VGG16 with pretrained parameters, Transfer Network based on ResNet50 with pretrained parameters, and Multitask Network based on VGG16 or ResNet50. Model or hyperparameters were adjusted constantly to obtain a better model. According to the rule of high accuracy and good stability in the labeled testing dataset, the optimal model was chosen as a PL prediction model. PL was generated again to form a PL dataset.

In the process of data cotraining, PL dataset was taken as one task, and the training dataset was taken as another task. The cotraining was the multitask training network with high similar task. If the optimal model in data cotraining had higher accuracy and better stability than that in the previous optimal model, the optimal model would be updated. The steps above were repeated several times until the end condition that the accuracy could not be improved was satisfied. In the process of iterative training, we find the best model with high accuracy and good stability, and the network gradually improved the accuracy of the main task. The testing dataset was used as the benchmark to test the accuracy of the task. The dispersion degree of the accuracy of multiple experimental results was used as the benchmark to measure the stability of the model.

The article "Application Research for Fusion Model of Pseudolabel and Cross Network" was published in 2022. Journal: Comput Intell Neurosci.

### 2.4. Implementation of Fusion Model of PL and CN

In MTL, the common methods include parameter hard sharing mechanism and parameter soft sharing mechanism [17]. In the parameter hard sharing mechanism, there is same feature sharing layer, and the task-independent feature layer is retained, which greatly reduced the risk of overfitting. The sharing structure was easy to understand and implement. It was an effective way, but was a “rude” way of parameter sharing. In parameter soft sharing mechanism, there was a kind of sharing based on constraints, in which each task had its own feature parameters and constraints between tasks. This design was more robust than parameter hard sharing mechanism, and there were many ways to implement it. In soft sharing mechanism, parameters were shared between layers according to certain rules and strategies.

Figure 5 showed the implementation of fusion model of PL and CN. Among them, two different inputs corresponded to Net1 and Net2 subnetworks. Two subnetworks were trained, respectively, and combined into a MTL network by Cross Unit, in which the parameters could be shared according to the needs. Cross Unit between two subnetworks was like a “valve” controlling the network sharing degree. In Figure 5, Net1 and Net2 were used to learn the mapping from feature space to real labeled space and from feature space to PL space, respectively. The network used some real labeled dataset to assist network training. PL was applied to supervise Net1 network, and the real label to supervise Net2 network. Classifier 1 and Classifier 2 were trained through PL data and labeled training dataset, respectively.

In MTL, CN was applied [11]. By activating multiple networks, End-to-End Learning was carried out. Then, the sharing layer was automatically determined, which was the best combination of shared features, and independent features representation could be learned from networks of Cross Unit. Firstly, PL dataset and the original dataset were preprocessed. Secondly, the data were input into two subnetworks for training, in which the subnetworks shared parameters through Cross Unit. Finally, Classifier 1 and Classifier 2 were obtained.

The weight of the multitask loss function was expressed as

(1) $$\begin{array}{c} L_{\text{total}}=\sum_{t=1}^{T}\omega_{t}*L_{t}. \end{array}$$

Here *L*_total_ represented the total loss of the model, *L*_*t*_ represented the loss of the *t*th task, *ω*_*t* _ represented the corresponding weight of the *t*th task, and *T*  represented the number of tasks trained by the model.

The article "Application Research for Fusion Model of Pseudolabel and Cross Network" was published in 2022. Journal: Comput Intell Neurosci.

Assume that the activation maps of two tasks are  *x*_1_ and *x*_2_ , features of the linear combination of two input activation maps are ${\tilde{x}}_{1}$ and ${\tilde{x}}_{2}$. Suppose that *α*_12_ and *α*_21_ represent the weight between different tasks, *α*_11_ and *α*_22_ represent the weight between the same tasks. The weight matrix encoded the relationship between two tasks, and *α*_12_, *α*_21_, *α*_11_, and *α*_22_ could be set to adjust sharing degree. The linear combination of the activation maps was used as the input of the next layer network. Adjusting the values of *α*_12_ , *α*_21_ , *α*_11_, and *α*_22_ can optimize the linear combination of the activation maps. *α*_12 _  or  *α*_21 _  could be set to 0 for training of tasks; there was no shared feature between the two networks. *α*_11_ or *α*_22_ could be set to 1 for training of tasks; all parameters between the two networks were shared. Hyperparameters could be assigned different values to represent different sharing degrees. The calculation formula of Cross Unit could be expressed as

(2) $$\begin{array}{c} \left[\begin{array}{c} {\tilde{x}}_{1}\\ {\tilde{x}}_{2} \end{array}\right]=\left[\begin{array}{c} \alpha_{11}\\ \alpha_{21} \end{array}\right)\left(\begin{array}{c} \alpha_{12}\\ \alpha_{22} \end{array}\right]\left[\begin{array}{c} x_{1}\\ x_{2} \end{array}\right]. \end{array}$$

## 3. Experimental Results and Analysis

### 3.1. Experimental Basis

Experiment adopted AMD computer processor with six cores and twelve threads. The capacity of the graphics card GeForce RTX 2080 was 8G. Motherboard memory capacity was 32G. PyTorch was adopted as deep learning framework. GPU parallel computing architecture was CUDA Toolkit 10.0, and cuDNN based on CUDA was 7.5. Python version was 3.6, and so on.

### 3.2. Experimental Objects and Processing

The SCUT-FBP5500 dataset, Fer2013 dataset, Large-Scale Asia Facial Beauty (LSAFB) dataset, and FaceShape dataset were applied in this paper.

#### 3.2.1. SCUT-FBP5500 Dataset

SCUT-FBP5500 dataset [18, 19], released by Human Computer Intelligent Interaction Laboratory of South China University of Technology, contained 5500 facial images, including 2000 Asian female, 2000 Asian male, 750 Caucasian female, and 750 Caucasian male. The dataset folder contained images and labels. According to the label of dataset, the image was divided into gender dataset, including training dataset and testing dataset. Then, the training dataset and testing dataset were divided into subfolders 0 and 1, where female images were stored in subfolder 0, male images were stored in subfolder 1, and the image size was changed. The processed dataset was regarded as Gender Recognition Dataset.

The article "Application Research for Fusion Model of Pseudolabel and Cross Network" was published in 2022. Journal: Comput Intell Neurosci.

#### 3.2.2. Fer2013 Dataset

Fer2013 dataset [20] was a commonly used expression recognition dataset, which was composed of 35,886 facial expression images, including 28,708 training images and 7178 testing images. Each image consisted of 48 × 48 gray image, with a total of seven kinds of expressions: anger, disgust, fear, happy, sad, surprised, and neutral, corresponding to digital labels 0–6, respectively. Firstly, the toolkit was used to read the dataset, and the Pixels, Emotion and Usage were obtained. Secondly, the training dataset and testing dataset were divided. Finally, the original image was saved in JPG format, classified according to label, and saved as the corresponding folder, respectively. The processed Fer2013 dataset was regarded as expression dataset.

#### 3.2.3. LSAFB Dataset

LSAFB Dataset [21] was constructed by our Project Team, including 20,000 labeled images and 80,000 unlabeled images, with a total of 100,000 images. 10,000 label images of female were regarded as experimental dataset. Good results on this dataset was achieved in [22]. Facial beauty images can be divided into five categories: extremely unattractive, unattractive, medium, attractive, and extremely attractive, corresponding to digital labels 0–4, respectively. There are 948 images in the “0” category, 1148 images in the “1” category, 3846 images in the “2” category, 2718 images in the “3” category, and 1340 images in the “4” category. LSAFB dataset was divided into training dataset and testing dataset according to the label. In the process of data training, the images of each subfolder were read, changed to the specified size, and the data was scrambled at the same time. The processed LSAFB dataset was regarded as Facial Beauty Dataset.

#### 3.2.4. FaceShape Dataset

FaceShape Dataset [23] was composed of 5000 female celebrity images all over the world, with storage capacity of 694M. It was released by Machine Learning enthusiasts on the data science competition platform—Kaggle. According to the shape of faces, the images were divided into five categories: heart, rectangle, ellipse, circle, and square. The dataset was divided into various categories, and each category contained 1000 images. This dataset could be used to train neural networks with different facial features. Network input required a fixed size, so uniform size processing was performed. The dataset was regarded as Unlabeled Facial Dataset.

### 3.3. Model Evaluation and Analysis

Table 1 showed experimental results of Facial Beauty Prediction in PL data generation part. Among them, VGG16, ResNet50, Transfer Network based on VGG16 with pretrained parameters, Transfer Network based on ResNet50 with pretrained parameters were all single-task networks, and the network input data was the training dataset. From the dimension of resolution, the accuracy with the resolution of 128 × 128 was higher and relatively stable. From the dimension of learning rate, the accuracy with learning rate of 0.003 was higher and relatively stable. Therefore, the hyperparameter model with the resolution of 128 × 128 and learning rate of 0.003 was chosen as the optimal model for PL generation. Then, PL was generated to prepare data for the next part.

The article "Application Research for Fusion Model of Pseudolabel and Cross Network" was published in 2022. Journal: Comput Intell Neurosci.

Table 2 showed experimental results of Facial Beauty Prediction in data cotraining part. Among them, VGG16, ResNet50, Transfer Network based on VGG16 with pretrained parameters, and Transfer Network based on ResNet50 with pretrained parameters were all single-task network. The input data of the network was the corresponding categories of training dataset and PL dataset. The input data from Multitask Network based on VGG16 and Multitask Network based on ResNet50 was training dataset and PL dataset. Every subnetwork was trained respectively, and the two subnetworks were combined into a Multitask Learning Network through Cross Unit. From the dimension of resolution, image with the resolution of 100 × 100 was performed well and stable in VGG16, ResNet50, Transfer Network based on VGG16 with pretrained parameters, and Transfer Network based on ResNet50 with pretrained parameters, while image with the resolution of 128 × 128 was performed well and stable in Multitask Network based on VGG16 or ResNet50. From the dimension of learning rate, learning rate of 0.003 was good and stable in VGG16, ResNet50, Transfer Network based on VGG16 with pre-trained parameters, and Transfer Network based on ResNet50 with pretrained parameters, and learning rate of 0.001 was good and stable in Multitask Network based on VGG16 and Multitask Network based on ResNet50. Therefore, the resolution of 100 × 100 and learning rate of 0.003 were good and stable in VGG16, ResNet50, Transfer Network based on VGG16 with pretrained parameters, and Transfer Network based on ResNet50 with pretrained parameters, and the resolution of 128 × 128 and learning rate of 0.001 were good and stable in Multitask Network based on VGG16 and Multitask Network based on ResNet50. Experiments show that when the learning rate was small, experimental result was better, but it should not be too small; otherwise, the training time will be greatly increased. The closer the original resolution, the better experimental results. In order to speed up the training speed and reduce the complexity of the model, we can appropriately reduce the resolution and make trade-offs between efficiency and results. Multitask network was better than single-task network. The Multitask Network based on VGG16 performed better, which could be chosen as the optimal model of PL generation to prepare for the next part of training. The steps above were repeated several times.

The article "Application Research for Fusion Model of Pseudolabel and Cross Network" was published in 2022. Journal: Comput Intell Neurosci.

In Table 3, Facial Beauty Prediction task and Gender Recognition task, Facial Beauty Prediction task and Expression Recognition task were trained on real labeled datasets, and the tasks with real label belonged to SL tasks. Multitask network used CN, and single-task network was VGG16 network. Single-task accuracy of Facial Beauty Prediction was 58.75%. In the CN of MTL, the highest accuracy of main task of Facial Beauty Prediction was 64.06%. This strongly proved that MTL could greatly improve the accuracy of main task. By adjusting the hyperparameters *α*, different hyperparameters *α* would lead to different accuracy of main task, which proved that the hyperparameters *α* could adjust the sharing degree of the network, and it was a more effective adjustable way.

In Table 4, multitask network was trained on Facial Beauty Dataset with real label, and the task with real label belonged to SL task, while multitask network was trained on FaceShape Dataset with PL, and the task with PL belonged to WSL task. Multitask network was a CN based on VGG16 and ResNet50, and single-task network was VGG16. In Table 4, the constraint rule of regular hyperparameters *α* was *α*_11_+*α*_12_=1, and the diagonal value was equal and the value was positive. In Facial Beauty Dataset and FaceShape Dataset, the regular hyperparameters *α* were adjusted continuously. The single-task accuracy of Facial Beauty Prediction was 58.75%. In the CN based on VGG16 and ResNet50, the highest accuracy of the main task of Facial Beauty Prediction was 62.95%.

In Facial Beauty Dataset and FaceShape Dataset, the irregular hyperparameters *α* were adjusted continuously and the following rules were observed: 0 < *α*_11_ < 1,0 < *α*_12_ < 1. In the meantime, diagonal values were equal, and the values were all positive.

As can be seen from Table 5, when the network performance of the task was good, the hyperparameters *α* were not higher than 0.5. Thus, the task sharing degree was not high, and the accuracy of facial beauty prediction task was up to 64.76%. In fact, it was related to the data. The similarity between faces was relatively high, and the similarity between faces of adjacent categories was higher, so it was difficult to distinguish their categories. Due to different datasets, there were differences in data distribution. The fusion of FaceShape Dataset and Facial Beauty Dataset will bring a certain amount of noise. To a certain extent, the noise data will improve the generalization ability of the model, but the noise data beyond a certain limit will lead to the deviation of the learning direction of the model and cannot correctly learn the information of the image itself so that the accuracy of the model is reduced, or even the accuracy fluctuates greatly.

The article "Application Research for Fusion Model of Pseudolabel and Cross Network" was published in 2022. Journal: Comput Intell Neurosci.

It can be seen from Tables 2–4 that different network structures, different data, and different tasks may result in different hyperparameters with excellent performance, and the specific values of hyperparameters need be determined through more experiments. It can be seen from Table 3 that SL improved the task of Facial Beauty Prediction to 64.06%. From Table 5, it can be seen that PL data improved the task of Facial Beauty Prediction to 64.76%. PL can improve main task of Facial Beauty Prediction compared with SL task, and slightly higher than the highest accuracy of SL. This strongly proved the effectiveness of PL.

## 4. Conclusion and Prospect

In the experiments of the fusion model of PL and CN, Facial Beauty Prediction was regarded as main task and the others as auxiliary tasks. It was suitable for multitask training of different tasks in different or similar datasets. The model achieved good experimental results on main task of Facial Beauty Prediction. In the fusion model of PL and CN, PL was applied to make better use of a large number of unlabeled data in PL data generation part; CN was applied to realize parameter sharing between layers and modules in data cotraining part. SL improved the main task of Facial Beauty Prediction by 64.06%, and PL data improved the main task of Facial Beauty Prediction by 64.76%. In Facial Beauty Prediction task, PL was more effective than SL, which will greatly promote the application of PL in a wider range of fields. But there were also some problems of low accuracy in some experiments. In the future, Generative Adversarial Network will be applied in WSL, and the method of fitting data residual method will be used to continuously improve the performance of the algorithm.

## Figures and Tables

**Figure 1:** Block diagram of fusion model of PL and CN.

**Figure 2:** Block diagram of data preprocessing.

**Figure 3:** Block diagram of PL data generation.

**Figure 4:** Block diagram of data cotraining.

**Figure 5:** Fusion model of PL and CN structure diagram.

**Table 1:** Experimental results of PL generation part.

Hyperparameters		Model			
		VGG16 [11]	ResNet50 [12] (%)	Transfer network	
				VGG16 (%)	ResNet50 (%)
Resolution	32 × 32	53.06	48.34	53.56	53.16
	64 × 64	53.36	53.36	53.51	54.57
	72 × 72	54.02	53.71	53.71	52.46
	96 × 96	53.16	54.27	55.12	54.72
	100 × 100	58.84	55.47	54.82	54.92
	**128** × **128**	**60.43**	**58.33**	**60.34**	**58.84**

Learning rate	0.001	53.51	53.97	53.16	52.06
	**0.003**	**60.43**	**58.33**	**60.34**	**58.84**
	0.01	53.12	54.02	54.07	53.66
	0.03	56.12	52.51	54.47	53.82
	0.1	44.28	54.07	53.56	53.31
	0.3	44.18	44.28	44.78	44.43

Better results in terms of recognition rates were highlighted in bold.

The article "Application Research for Fusion Model of Pseudolabel and Cross Network" was published in 2022. Journal: Comput Intell Neurosci.

**Table 2:** Experimental results of cotraining part.

Hyperparameters		Model					
		VGG16 [11]	ResNet50 [12] (%)	Transfer network		Multitask network	
				VGG16 (%)	ResNet50 (%)	VGG16 (%)	ResNet50 (%)
Revolution	32 × 32	56.04	52.45	53.15	54.55	60.94	60.29
	64 × 64	55.36	53.36	55.44	54.34	61.10	60.80
	72 × 72	56.37	54.71	53.71	54.59	60.25	60.10
	96 × 96	55.22	54.20	55.12	55.42	60.94	60.60
	**100** **×** **100**	**61.38**	**59.34**	**61.29**	**59.47**	60.10	57.43
	**128** **×** **128**	59.66	56.65	55.87	54.86	**61.45**	**60.74**

Learning rate	**0.001**	56.74	55.56	55.11	54.27	**61.95**	**61.50**
	**0.003**	**61.38**	**59.34**	**61.29**	**59.47**	60.10	57.43
	0.01	56.07	55.05	56.37	55.74	55.82	59.74
	0.03	57.42	54.49	56.65	56.57	54.02	50.64
	0.1	46.18	55.32	55.44	55.37	48.36	48.44
	0.3	48.23	46.53	47.61	45.46	47.98	45.55

Better results in terms of recognition rates were highlighted in bold.

**Table 3:** Experimental results of multitask and single task.

(*α*_11_, *α*_12_, *α*_21_, *α*_22_)	Multitask		Multitask		Single task
	Facial beauty prediction (%)	Gender recognition (%)	Facial beauty prediction (%)	Expression recognition (%)	Facial beauty prediction (%)
(0, 1, 1, 0)	60.94	97.64	63.35	23.99	**58.75**
(0.1, 0.9, 0.9, 0.1)	62.85	96.91	62.55	45.91	
(0.2, 0.8, 0.8, 0.2)	**64.06**	95.64	62.45	49.85	
(0.3, 0.7, 0.7, 0.3)	62.65	97.82	62.95	38.95	
(0.4, 0.6, 0.6, 0.4)	—	55.82	61.75	44.85	
(0.5, 0.5, 0.5, 0.5)	61.65	95.45	62.75	32.80	
(0.6, 0.4, 0.4, 0.6)	62.35	94.73	62.65	45.67	
(0.7, 0.3, 0.3, 0.7)	61.55	95.82	63.45	46.21	
(0.8, 0.2, 0.2, 0.8)	62.85	96.55	61.35	48.91	
(0.9, 0.1, 0.1, 0.9)	63.45	96.55	62.35	47.94	
(1, 0, 0, 1)	59.35	97.45	63.05	23.99	

Better results in terms of recognition rates were highlighted in bold.

**Table 4:** Experimental results of regular hyperparameters *α* values.

(*α*_11_, *α*_12_, *α*_21_, *α*_22_)	VGG16 of CN [11]		ResNet50 of CN [12]		Single-task
	Facial Beauty dataset (%)	FaceShape dataset (%)	Facial Beauty dataset (%)	FaceShape dataset (%)	Facial Beauty Prediction (%)
(0, 1, 1, 0)	—	56.65	—	57.40	**58.75**
(**0.1, 0.9, 0.9, 0.1**)	62.35	58.91	**62.95**	56.35	
(0.2, 0.8, 0.8, 0.2)	62.25	57.65	61.70	57.20	
(0.3, 0.7, 0.7, 0.3)	62.25	56.85	62.60	57.45	
(0.4, 0.6, 0.6, 0.4)	62.10	56.80	62.40	57.40	
(0.5, 0.5, 0.5, 0.5)	61.80	57.05	61.55	56.80	
(0.6, 0.4, 0.4, 0.6)	62.30	57.35	62.50	57.25	
(0.7, 0.3, 0.3, 0.7)	62.40	57.60	62.05	57.90	
(0.8, 0.2, 0.2, 0.8)	62.30	57.45	62.90	58.71	
(0.9, 0.1, 0.1, 0.9)	62.80	57.10	62.70	58.20	
(1, 0, 0, 1)	61.19	57.20	—	57.95	

Better results in terms of recognition rates were highlighted in bold.

The article "Application Research for Fusion Model of Pseudolabel and Cross Network" was published in 2022. Journal: Comput Intell Neurosci.

**Table 5:** Experimental results of irregular hyperparameters *α* values.

(*α*_11_, *α*_12_, *α*_21_, *α*_22_)	Facial Beauty Prediction (%)	(*α*_11_, *α*_12_, *α*_21_, *α*_22_)	Facial Beauty Prediction (%)	(*α*_11_, *α*_12_, *α*_21_, *α*_22_)	Facial Beauty Prediction (%)
(0.1, 0.1, 0.1, 0.1)	62.55	(0.4, 0.1, 0.1, 0.4)	62.55	(0.7, 0.1, 0.1, 0.7)	63.21
(0.1, 0.2, 0.2, 0.1)	62.45	(**0.4, 0.2, 0.2, 0.4**)	**64.11**	(0.7, 0.2, 0.2, 0.7)	62.70
(0.1, 0.3, 0.3, 0.1)	62.25	(**0.4, 0.3, 0.3, 0.4**)	**63.00**	(0.7, 0.3, 0.3, 0.7)	63.16
(0.1, 0.4, 0.4, 0.1)	63.10	(**0.4, 0.4, 0.4, 0.4**)	**64.76**	(0.7, 0.4, 0.4, 0.7)	62.60
(0.1, 0.5, 0.5, 0.1)	64.66	(**0.4, 0.5, 0.5, 0.4**)	**63.20**	(0.7, 0.5, 0.5, 0.7)	62.65
(0.1, 0.6, 0.6, 0.1)	62.95	(0.4, 0.6, 0.6, 0.4)	62.35	(0.7, 0.6, 0.6, 0.7)	62.00
(0.1, 0.7, 0.7, 0.1)	62.55	(0.4, 0.7, 0.7, 0.4)	62.60	(0.7, 0.7, 0.7, 0.7)	60.29
(0.1, 0.8, 0.8, 0.1)	62.60	(0.4, 0.8, 0.8, 0.4)	—	(0.7, 0.8, 0.8, 0.7)	—
(0.1, 0.9, 0.9, 0.1)	63.15	(0.4, 0.9, 0.9, 0.4)	62.10	(0.7, 0.9, 0.9, 0.7)	—
(0.2, 0.1, 0.1, 0.2)	62.15	(0.5, 0.1, 0.1, 0.5)	63.15	(0.8, 0.1, 0.1, 0.8)	62.50
(0.2, 0.2, 0.2, 0.2)	62.55	(0.5, 0.2, 0.2, 0.5)	63.56	(0.8, 0.2, 0.2, 0.8)	62.55
(0.2, 0.3, 0.3, 0.2)	62.42	(0.5, 0.3, 0.3, 0.5)	63.00	(0.8, 0.3, 0.3, 0.8)	63.20
(0.2, 0.4, 0.4, 0.2)	62.85	(0.5, 0.4, 0.4, 0.5)	61.50	(0.8, 0.4, 0.4, 0.8)	63.30
(0.2, 0.5, 0.5, 0.2)	62.70	(0.5, 0.5, 0.5, 0.5)	62.20	(0.8, 0.5, 0.5, 0.8)	—
(0.2, 0.6, 0.6, 0.2)	62.28	(0.5, 0.6, 0.6, 0.5)	63.15	(0.8, 0.6, 0.6, 0.8)	60.74
(0.2, 0.7, 0.7, 0.2)	61.10	(0.5, 0.7, 0.7, 0.5)	62.80	(0.8, 0.7, 0.7, 0.8)	63.38
(0.2, 0.8, 0.8, 0.2)	62.55	(0.5, 0.8, 0.8, 0.5)	62.85	(0.8, 0.8, 0.8, 0.8)	62.35
(0.2, 0.9, 0.9, 0.2)	62.70	(0.5, 0.9, 0.9, 0.5)	61.24	(0.8, 0.9, 0.9, 0.8)	62.80
(0.3, 0.1, 0.1, 0.3)	61.55	(0.6, 0.1, 0.1, 0.6)	63.05	(0.9, 0.1, 0.1, 0.9)	63.10
(0.3, 0.2, 0.2, 0.3)	62.80	(0.6, 0.2, 0.2, 0.6)	62.75	(0.9, 0.2, 0.2, 0.9)	63.00
(0.3, 0.3, 0.3, 0.3)	62.40	(0.6, 0.3, 0.3, 0.6)	63.26	(0.9, 0.3, 0.3, 0.9)	62.40
(0.3, 0.4, 0.4, 0.3)	62.95	(0.6, 0.4, 0.4, 0.6)	62.60	(0.9, 0.4, 0.4, 0.9)	62.20
(0.3, 0.5, 0.5, 0.3)	63.76	(0.6, 0.5, 0.5, 0.6)	63.20	(0.9, 0.5, 0.5, 0.9)	63.71
(0.3, 0.6, 0.6, 0.3)	63.56	(0.6, 0.6, 0.6, 0.6)	62.68	(0.9, 0.6, 0.6, 0.9)	—
(0.3, 0.7, 0.7, 0.3)	62.32	(0.6, 0.7, 0.7, 0.6)	61.60	(0.9, 0.7, 0.7, 0.9)	—
(0.3, 0.8, 0.8, 0.3)	62.45	(0.6, 0.8, 0.8, 0.6)	—	(0.9, 0.8, 0.8, 0.9)	62.39
(0.3, 0.9, 0.9, 0.3)	62.30	(0.6, 0.9, 0.9, 0.6)	—	(0.9, 0.9, 0.9, 0.9)	—

Better results in terms of recognition rates were highlighted in bold.

The article "Application Research for Fusion Model of Pseudolabel and Cross Network" was published in 2022. Journal: Comput Intell Neurosci.

## Data Availability

The data used to support the findings of this study are available from the corresponding author upon request or are from previously reported studies and datasets, which have been cited.
